# Circular RNA CircSHKBP1 accelerates the proliferation, invasion, angiogenesis, and stem cell-like properties via modulation of microR-766-5p/high mobility group AT-hook 2 axis in laryngeal squamous cell carcinoma

**DOI:** 10.1080/21655979.2022.2068922

**Published:** 2022-05-03

**Authors:** Fu Chen, Haiyan Zhang, Jie Wang

**Affiliations:** Department of Radiation Oncology, Eye & ENT Hospital of Fudan University, Shanghai, China

**Keywords:** CircSHKBP1, MiR-766-5p, HMGA2, tumorigenesis, laryngeal squamous cell carcinoma

## Abstract

Laryngeal squamous cell carcinoma (LSCC) is a common malignancy in head and neck. Circular SHKBP1 (circSHKBP) exerts momentous functions in the occurrence of many cancers including LSCC. Thus, we investigated the oncogenic capacities of circSHKBP1 in LSCC, and revealed the underlying mechanism as a competing endogenous RNA. The expression levels of circSHKBP1, miR-766-5p, and high mobility group AT-hook 2 (HMGA2) were examined by quantitative real-time PCR and their influences on the overall survival were measured by Kaplan–Meier method. The correlations between circSHKBP1 and miR-766-5p or HMGA2 were detected by Spearman’s rank correlation analysis. *In vitro*, the influences of circSHKBP1/miR-766-5p/HMGA2 axis on the tumorigenesis of LSCC were examined by CCK-8, transwell, sphere formation, and angiogenesis assays, respectively. circSHKBP1 expression was up-regulated in the LSCC specimens and cell lines. And elevated circSHKBP1 expression was closely linked to poor prognosis. Silencing circSHKBP1 expression restrained cell proliferation, invasion, angiogenesis, stem cell-like properties and tumor growth. We observed that miR-766-5p was down-regulated and negatively correlated to circSHKBP1 in LSCC samples. However, HMGA2 was highly expressed and positively associated with circSHKBP1 in these specimens. Importantly, the levels of circSHKBP1, miR-766-5p, and HMGA2 were closely associated with patients’ clinical parameters including lymph nodes metastasis and TNM stages. Mechanistic analysis clarified that circSHKBP1 sponged miR-766-5p to regulate HMGA2, the target of miR-766-5p. Moreover, miR-766-5p inhibition and overexpression of HMGA2 rescued the tumor-suppressing roles of circSHKBP1 downregulation in LSCC. In conclusion, circSHKBP1 accelerated the tumorigenesis of LSCC via modulating HMGA2 by targeting miR-766-5p.

## Highlights

- Increased circSHKBP1 expression indicates poor prognosis in patients with LSCC.
- Knockdown of circSHKBP1 expression suppresses malignant behaviors o LSCC cells.
- circSHKBP1 regulates LSCC tumorigenesis via miR-766-5p/HMGA2 axis.

## Introduction

Globally, almost 184,615 new cases of laryngeal cancer were diagnosed and 99,840 people die from this disease in 2020 [1]. As a frequent type of laryngeal cancer, laryngeal squamous cell carcinoma (LSCC) imposes a huge burden on patients and health system [2]. In spite of the advancement of treatment modality, we have not seen the obvious improvement of the 5-year survival rate of LSCC patients [3]. As with other tumors, the progression of LSCC is a complicated procedure that involves in alterations of metabolic, gene, and pathway [4,5]. Nevertheless, the pathogenesis of LSCC has not been defined clearly. Thus, clarifying the molecular mechanism of LSCC is eagerly needed.

Circular RNAs (circRNAs) exert momentous functions in the occurrence of many cancers including LSCC [6–8]. Previous study has stated that circRNAs regulated tumor development as competing endogenous RNAs (ceRNAs), that is, circRNAs functioned by sponging miRNAs to directly target mRNAs [9]. CircRNA-associated-ceRNA networks have been verified in the progression of LSCC. For instance, Tian et al. [10] have demonstrated that circRASSF2 accelerated LSCC progression via modulating miR-302b-3p/ insulin-like growth factor 1 receptor axis. The miR-223/ transforming growth factor beta receptor 3 axis was responsible for the tumorigenicity of circ0042666 in LSCC cells [11]. circPPFIA1 regulated the proliferation and migration of LSCC cells via sponging miR-340-3p [12].

CircSHKBP1 was highly expressed in the laryngeal cancer, which has been elucidated by RNA sequencing analysis in a previous study [13]. CircSHKBP1 has been demonstrated to facilitate angiogenesis and tumorigenicity in other cancers including glioma and gastric cancers [14,15]. miR-766-5p was deemed as a tumor-suppressing factor, which suppressed metastasis and promoted apoptosis of tumor cells [16–18]. High mobility group AT-hook 2 (HMGA2) has been reported to be up-regulated in LSCC and was relevant to patients’ poor prognosis [19]. Bioinformatic analysis displayed that there were complementary sequences between circSHKBP1 and miR-766-5p as well as between miR-766-5p and HMGA2. However, whether a ceRNA network exists among the three molecules is still unknown.

The current study aimed at exploring whether circSHKBP1-associated ceRNA network was implicated in LSCC progression. Our results demonstrated that circSHKBP1 was up-regulated in LSCC specimens and cell lines, and circSHKBP1 expression was strongly correlated with poor prognosis and clinical parameters, including lymph nodes metastasis and TNM stages, in LSCC. Moreover, circSHKBP1 modulated HMGA2 expression via targeting miR-766-5p, which implied new targets for LSCC therapy.

## Materials and methods

### Tissue specimens

60 LSCC patients who underwent surgery at Eye & ENT Hospital of Fudan University from January 2013 to December 2015 were enrolled in this study. Tissues including tumors and adjacent normal samples were obtained from these participants. Prior to surgery, all patients did not receive any chemotherapy or radiotherapy. These subjects have provided written informed consent. This study was approved by the Ethics Committee of the Eye & ENT Hospital of Fudan University (approval no. SYXK (沪) 2018–0019).

### Cell culture and transfection

16-HBE human bronchial epithelioid cells, human LSCC cell lines (TU686 and AMC-HN-8), and human umbilical vascular endothelial cells (HUVECs) were bought from Cell Resource Center, IBMS, CAMS/PUMC, where they were authenticated by short tandem repeat (STR) profiling. Conventional culture of all cells was performed using DMEM medium, which contains 10% fetal bovine serum (FBS) and 1% penicillin/streptomycin (BI, Israel). Upon reaching 80% confluence, LSCC cells were transfected with circSHKBP1 siRNA (si-circSHKBP1) or its control si-NC (Genechem, Shanghai, China) using Lipofectamine 2000. pcDNA-HMGA2 (HMGA2) and pcDNA-circSHKBP1 (circSHKBP1) overexpressing plasmids were synthesized by Genechem, whereas, miR-766-5p, miR-766-5p inhibitor, miR-NC, and NC inhibitor were from RiboBio (Guangzhou, China). To verify the stability of circSHKBP1, AMC-HN-8 cells were incubated with actinomycin D and RNase (Sigma, St. Louis, MO, USA), respectively.

### Quantitative real-Time PCR (qRT-PCR) assay

qRT-PCR experiment was performed according to a previous study [20]. After indicated treatments, cells and tissues were collected to extract total RNAs with Trizol reagent (CWBio, Beijing, China). qRT-PCR examination was carried out on TL988-II system (Tianlong, Xi’an, China) after synthesis of the first strand cDNA. Primers were listed in Table 1. The results were quantified by the 2-ΔΔCT method, in which β-actin or U6 was used as an internal control for circSHKBP1 and HMGA2, or miR-766-5p, respectively.

**Table 1.** Primer sequences

Gene	Forward (5’-3’)	Reverse (5’-3’)
circSHKBP1	AGGTCAGCAGAGGAAGTCA	CGCGTCATAACTGGTGATGG
HMGA2	CACATTTCAAGGGACAC	GCTGCCACCATCAACACC
β-actin	AGCGAGCATCCCCCAATT	GGGCACGAAGGCTCATCATT
miR-766-5p	TAGATAGAGACGTTCATA	ATACTATCTGGAGCTACA
U6	GCTCGCTTCGGCAGCACA	GAACGCTTCACGAATTTGCGTG

### CCK-8 assay

After transfection, LSCC cells (2 × 103 cells/well) were cultured at 37°C for 48 h. Afterward, cells were hatched for another 4 h after adding to CCK-8 solution (10 μL for each well). The absorbance at 450 nm was tested by a microplate reader (DNM-9606, Perlong, Beijing, China).

### Transwell assay for cell invasion

Transfected cells (2 × 10^4^ cells) were planted into the upper transwell chamber (8.0 µm pore size, Corning, Lowell, MA, USA), which was precoated by Matrigel, and the lower chamber was with 700 µL complete medium. 24 h later, the invasive cells were dyed with 0.1% crystal violet after removing cells remaining on the upper chamber, and fixing with 4% paraformaldehyde. Cell number was quantified under a microscope (CKX53, Olympus, Tokyo, Japan).

### Angiogenesis assay

The method for angiogenesis assay in vitro has been illustrated previously [21]. Briefly, LSCC cells were transfected with si-circSHKBP1, miR-766-5p, and HMGA2 for 24 h. After changing to serum-free DMEM medium, cells were hatched for another 48 h. Then, culture medium was obtained, centrifuged, and filtered to get tumor-conditioned medium. Subsequently, HUVECs (1 × 10^5^ cells/well) suspended in 100 μL tumor-conditioned medium were placed into the 96-well plates pre-coated with Matrigel and maintained at 37°C for 8 h. Tube formation was captured by a microscope (CKX53). Tube formation was quantified by measuring the total tubule length and number of tubule branches from five randomly selected fields.

### Sphere formation assay

Sphere formation of tumor cell in vitro was assayed in accordance with a previous study [22]. Transfected LSCC cells (1 × 10^3^ cells/well) were placed into ultra-low-attachment plates, and cultured in serum-free DMEM medium, which was supplemented with 20 ng/mL containing epidermal growth factor and 10 ng/mL basic fibroblast growth factor. After incubation for 10 days, the spheres were recorded under a microscope (CKX53).

### Dual-luciferase reporter assay

circSHKBP1-WT and circSHKBP1-MUT recombinant vectors were established by cloning the wild-type (WT) and mutant (MUT) fragments of circSHKBP1 into the pmirGLO vector. Correspondingly, the WT and MUT fragments of HMGA2 were subcloned into the pmirGLO vector to generate HMGA2-WT and HMGA2-MUT plasmids. These recombinant vectors and miR-766-5p were co-transfected into AMC-HN-8 cells for 48 h to detect luciferase activities.

### RNA pull-down assay

AMC-HN-8 cells were transfected with biotin-labeled circSHKBP1 probe or its control (Bio-NC) (RiboBio). 48 h later, cells were collected and lysed. The lysates were maintained with magnetic beads for 3 h, followed by purification. Then, the enrichment of miR-766-5p was examined by qRT-PCR assay.

### Western blotting assay

Proteins from cells were extracted using RIPA lysis buffer (Beyotime, Shanghai, China). After separating, isolated proteins were electrotransferred onto PVDF membranes. Next, 5% skimmed milk was used to block the membranes. Then, these membranes were incubated with primary antibodies including anti-HGMA2 (1:10,000, SAB2701959, Sigma, St. Louis, MO, USA), anti-proliferating cell nuclear antigen (PCNA) (1:2000, SAB5700622, Sigma), anti-matrix metallopeptidase 2 (MMP-2) (1:1000, SAB5700824, Sigma), anti-vascular endothelial growth factor A (VEGFA) (1:1500, SAB5700629, Sigma), and anti-POU class 5 homeobox 1 (POU5F1 or OCT4) (1:1000, SAB1306212, Sigma), and anti-β-actin (1:5000, 20,536-1-AP, Proteintech, Chicago, IL, USA). Behind that, membranes were hatched with HRP-conjugated secondary antibody (1:5000, ZB-2301, ZSGB, Beijing, China). Finally, a chemiluminescent imaging system (Tanon, Shanghai, China) was utilized to visualize protein bands, which were treated with enhanced chemiluminescence (ECL) kit.

### Tumorigenesis assay in vivo

5-week-old BALB/c nude mice were purchased from Hangzhou Ziyuan Laboratory Animal Science and Technology Co. Ltd (Hangzhou, China). These animals were assigned into sh-circSHKBP1 and sh-NC groups (n = 6 mice per group), which were inoculated with 200 μL of AMC-HN-8 cells (1 × 10^6^ cells/mL) transfected with sh-circSHKBP1 or sh-NC. From 1 week to 5 weeks, tumor volume was assessed once a week by the formula: Volume = (width) [2] × length/2. Mice were euthanized by intraperitoneally injection of pentobarbital sodium at day 35 after inoculation. The animal experiments were approved by the Animal Ethics Committee of Eye & ENT Hospital of Fudan University (approval no. SYXK (沪) 2018–0019).

### Immunohistochemistry

After fixating with 4% paraformaldehyde, tumor specimens of mice were dehydrated, and embedded into paraffin. Tissue blocks were cut into 5 µm slices. And each section was treated with 3% hydrogen peroxide in methanol, followed by blocking with 10% goat serum. Then, the slices were washed and incubated by anti-HMGA2 (1:500, SAB2701959), anti-PCNA (1:200, SAB5700622), MMP-2 (1:200, SAB5700824), VEGFA (1:100, SAB5700629), or OCT4 (1:50, SAB1306212) primary antibody overnight. After washing, HRP-labeled IgG secondary antibody (1:500, ZB-2301, ZSGB) was added to the samples. Subsequently, sections were stained with 3,3’-diaminobenzidine (ab64238, Abcam, MA, USA) and visualized by using a microscope (CKX53).

### Statistical analysis

SPSS 20.0 statistical software was used to analyze collected data. Differences in multiple groups were analyzed by one-way ANOVA followed by LSD test. The correlation between circSHKBP1 and miR-766-5p or HMGA2 was assayed by Spearman’s rank correlation analysis. The associations between circSHKBP1/miR-766-5p/HMGA2 and overall survival of LSCC patients were measured by Kaplan–Meier method with a log-rank test. *P* <0.05 was deemed as statistically significant.

## Results

The present study sought to investigate the expression and role of circSHKBP1 in LSCC. We found that circSHKBP1 expression was enhanced and negatively correlated with LSCC patients’ prognosis. circSHKBP1 played a role in cancer cell proliferation, invasion, angiogenesis and influenced stem cell-like properties. Mechanically, circSHKBP1 acted as a sponge of miR-766-5p and regulated HMGA2 expression in LSCC.

### CircSHKBP1 was up-regulated in LSCC and involved in patients’ poor prognosis

CircSHKBP1 expression was firstly tested in LSCC patients and cell lines to identify the impact of circSHKBP1 in LSCC. Results displayed that circSHKBP1 was up-regulated in 60 LSCC tissues in comparison with adjacent normal samples (*P* <0.001) (Figure 1a). We classified these patients into high circSHKBP1 group (n = 30) and low circSHKBP1 group (n = 30), according to the median expression of circSHKBP1. Patients with high circSHKBP1 expression showed lower overall survival (*P* <0.05) (Figure 1b). Also, circSHKBP1 expression was correlated with clinical parameters of LSCC patients including lymph nodes metastasis and TNM stages (Table 2). Consistently, circSHKBP1 levels in LSCC cells (TU686 and AMC-HN-8) were higher than that in 16-HBE cells (*P* <0.001) (Figure 1c). The structure of circSHKBP1 was shown in Figure 1d. The results of circSHKBP1 stability turned out that circSHKBP1 expression was not remarkably changed after exposure to actinomycin D and RNase, respectively (Figure 1e, 1f). The above mentioned findings indicated that circSHKBP1 was up-regulated in LSCC and involved in patients’ poor prognosis.

**Figure 1.** CircSHKBP1 was up-regulated in LSCC and involved in patients’ poor prognosis. (a) The circSHKBP1 expression in the 60 LSCC tissues and 60 adjacent normal samples (NC) was examined by qRT-PCR, ***P <0.001; (b) Kaplan–Meier method analysis for the influence of circSHKBP1 on the overall survival of LSCC patients; (c) qRT-PCR method for circSHKBP1 expression in TU686, AMC-HN-8 and 16-HBE cells, ***P <0.001, compared with 16-HBE cells; (d) The structure of circSHKBP1 was shown; (e and f) The stability of circSHKBP1 after exposure to actinomycin D and RNase was tested by qRT-PCR. **P <0.01, compared with GAPDH or Mock group. Experiments were conducted in triplicate. LSCC, laryngeal squamous cell carcinoma.

**Table 2.** Correlation between circSHKBP1 expression and the clinical pathological features of 60 LSCC patients

Characteristic	All cases	circSHKBP1 expression		P-value
		High (n = 30)	Low (n = 30)	
Gender				0.592
male	38	20	18	
female	22	10	12	
Age (years)				0.602
< 60	26	14	12	
≥60	34	16	18	
Smoking history				0.774
Nonsmokers	17	8	9	
Current smokers	43	22	21	
Lymph nodes metastasis				0.038*
Negative	32	12	20	
Positive	28	18	10	
TNM Stages				0.009*
I/II	28	9	19	
III/IV	32	21	11	

*P <0.05; LSCC, laryngeal squamous cell carcinoma.

### Silencing of circSHKBP1 restrained proliferation, invasion, angiogenesis, and stem cell-like properties of LSCC cells

*In vitro*, the influences of circSHKBP1 on the progression of LSCC were further investigated. As displayed in Figure 2a, circSHKBP1 expression in the si-circSHKBP1 groups, including si-circSHKBP1#1, si-circSHKBP1#2, and si-circSHKBP1#3, were notably decreased, compared with the si-NC group, with the lowest in the si-circSHKBP1#1 group. Thus, si-circSHKBP1#1 was chosen for the subsequent experiments. Silencing of circSHKBP1 effectively reduced cell viability (Figure 2b) and the number of invasive cells in TU686 and AMC-HN-8 cells (Figure 2c). Angiogenesis assay showed that the percentage of tube formation of HUVEC cells was sharply declined after treatment with tumor-conditioned medium from si-circSHKBP1-transfected LSCC cells (Figure 2d). CircSHKBP1-downregulating cells only formed 1/3-fold tumor spheres compared to the si-NC group (Figure 2e). Western blotting analysis demonstrated that silencing of circSHKBP1 outstandingly reduced the protein levels of PCNA, MMP2, VEGFA, and OCT4 (Figure 2f). However, we did not observe any changes of cell viability and expression of PCNA, MMP2, VEGFA, and OCT4 in circSHKBP1-silencing 16-HBE cells (**Supplemental Figure 1A-1C**). Taken together, these data indicated that si-circSHKBP1 restrained proliferation, invasion, angiogenesis, and stem cell-like properties of LSCC cells.

**Figure 2.** Silencing of circSHKBP1 restrained proliferation, invasion, angiogenesis and stem cell-like properties of LSCC cells. (a) Transfection efficacy of circSHKBP1 siRNA in cells was examined by qRT-PCR; (b) Cell viability was measured by CCK-8 assay; (c) The invasive ability of TU686 and AMC-HN-8 cells was measured by transwell assay after transfecting with si-circSHKBP1; (d) The percentage of tube formation of HUVEC cells treated with tumor-conditioned medium from si-circSHKBP1-transfected LSCC cells was shown; (e) Sphere formation assay for stem cell-like properties; (f) Levels of indicated proteins (PCNA, MMP2, VEGFA, and OCT4) were examined by western blotting. *P <0.05, **P <0.01, ***P <0.001, compared with si-NC group. Experiments were conducted in triplicate.

### CircSHKBP1 sponged miR-766-5p

Whether circSHKBP1 could deem as sponges for miRNAs in LSCC was proved in the current study. Starbase 3.0 software predicted that complementary binding sites were existed between circSHKBP1 and miR-766-5p (Figure 3a). Hence, we further investigated the relationship between circSHKBP1 and miR-766-5p in LSCC. In LSCC specimens, miR-766-5p expression was down-regulated (*P* <0.001) (Figure 3b), and its expression was involved in clinical parameters including lymph nodes metastasis and TNM stages (Table 3). What’s more, circSHKBP1 expression was negatively relevant to miR-766-5p level (r = −0.6196, *P* <0.001) (Figure 3c). Beyond that, a shorter overall survival was found in miR-766-5p-low-expressed patients (Figure 3d). Compared with 16-HBE cells, miR-766-5p expression in LSCC cells (Figure 3e). miR-766-5p outstandingly suppressed the relative luciferase activity of circSHKBP1-WT (*P* <0.01), but did not change that of circSHKBP1-MUT (Figure 3f). RNA pull-down results showed that the enrichment of miR-766-5p in bio-circSHKBP1 group was increased compared to the bio-NC group (*P* <0.001) (Figure 3g). Furthermore, miR-766-5p expression was prominently elevated by si-circSHKBP1 (Figure 3h). All aforementioned results suggested that circSHKBP1 could bind to miR-766-5p.

**Figure 3.** CircSHKBP1 sponged miR-766-5p. (a) The complementary binding sites of circSHKBP1 and miR-766-5p were predicated by Starbase 3.0; (b) MiR-766-5p expression in 60 LSCC tissues was lower than the adjacent normal (NC) samples, ***P <0.001; (c) The correlation between circSHKBP1 and miR-766-5p in LSCC samples; (d) The association between miR-766-5p and overall survival of LSCC patients was analyzed; (e) miR-766-5p expression in cells was tested by qRT-PCR, ***P <0.001, compared with 16-HBE cells; (f) Relative luciferase activity in AMC-HN-8 cells under different treatments was measured, **P <0.01, compared with miR-NC group; (g) RNA pull-down assay for the direct binding relationship between circSHKBP1 and miR-766-5p in AMC-HN-8 cells, ***P <0.001, compared with Bio-NC group; (h) miR-766-5p expression in si-circSHKBP1-transfected AMC-HN-8 cells; **P <0.01, compared with si-NC group. Experiments were conducted in triplicate. LSCC, laryngeal squamous cell carcinoma.

**Table 3.** Correlation between miR-766-5p expression and the clinical pathological features of 60 LSCC patients

Characteristic	All cases	miR-766-5p expression		P-value
		High (n = 30)	Low (n = 30)	
Gender				0.284
male	38	17	21	
female	22	13	9	
Age (years)				0.297
< 60	26	15	11	
≥60	34	15	19	
Smoking history				0.390
Nonsmokers	17	10	7	
Current smokers	43	20	23	
Lymph nodes metastasis				0.002*
Negative	32	22	10	
Positive	28	8	20	
TNM Stages				0.038*
I/II	28	18	10	
III/IV	32	12	20	

*P <0.05; LSCC, laryngeal squamous cell carcinoma.

### HMGA2 was the target of miR-766-5p and circSHKBP1 positively modulated HMGA2 expression via miR-766-5p

In the following, we analyzed whether a ceRNA network based on circSHKBP1 and miR-766-5p existed in LSCC. Starbase 3.0 software revealed that the 3’-UTR of HMGA2 contained a putative targeting site for miR-766-5p (Figure 4a). The relative luciferase activity of HMGA2-WT was remarkably reduced by miR-766-5p; however, miR-766-5p could not alter the relative luciferase activity of HMGA2-MUT, which were demonstrated by dual-luciferase reporter assay (Figure 4a). Beyond that, miR-766-5p overexpression lowered HMGA2 level, which was observed in Figure 4b. To validate the influences of circSHKBP1 and miR-766-5p on HMGA2, we firstly detected the transfection efficacy, and it turned out that miR-766-5p level was lower in miR-766-5p inhibitor group than that its control (*P* <0.001) (Figure 4c). Western blotting assay displayed that si-circSHKBP1 reduced HMGA2 expression, which was abrogated by miR-766-5p inhibitor (Figure 4d). We also found that upregulation of circSHKBP1 significantly increased HMGA2 expression in miR-766-5p highly expressed LSCC cells, but not in miR-766-5p-knockout cells (**Supplemental Figure 2**). *In vivo*, HMGA2 was highly expressed in LSCC specimens in contrast to adjacent normal samples, and high expression of HMGA2 was negatively relevant to patients’ poor prognosis (Figure 4e, 4f). The expression of HMGA2 was related to patients’ clinical parameters including lymph nodes metastasis and TNM stages (Table 4). Furthermore, HMGA2 expression was negatively associated with miR-766-5p level (r = 0.5931, *P* <0.001). Whereas a positive correlation was shown in the expression of HMGA2 and circSHKBP1 (r = 0.6559, *P* <0.001) (Figure 4g, 4h). *In vitro*, HMGA2 levels in LSCC cells were elevated in comparison with 16-HBE cells (*P* <0.05) (Figure 4i). These findings indicated that HMGA2 was the target of miR-766-5p and circSHKBP1 regulated HMGA2 by miR-766-5p instead of direct regulation.

**Figure 4.** HMGA2 was the target of miR-766-5p. (a) The targeting relationship between miR-766-5p and HMGA2 was predicated by Starbase 3.0 and examined by dual-luciferase reporter assay; (b) miR-766-5p decreased HMGA2 protein level in AMC-HN-8 cells, **P <0.01, compared with miR-NC group; (c) Transfection efficacy of miR-766-5p inhibitor was determined in AMC-HN-8 cells, **P <0.01, compared with miR-NC group; (d) HMGA2 protein level in AMC-HN-8 cells transfecting with si-circSHKBP1, or si-circSHKBP1 and miR-766-5p inhibitor, **P <0.01, ***P <0.001; (e) qRT-PCR assay for HMGA2 expression in LSCC specimens, ***P <0.001; (f) High expression of HMGA2 was associated with LSCC patients’ shorter overall survival; (g, h) The association between HMGA2 and miR-766-5p or circSHKBP1 in LSCC patients; (i) HMGA2 protein levels in both LSCC cells, *P <0.05, **P <0.01, compared with 16-HBE cells. Experiments were conducted in triplicate. LSCC, laryngeal squamous cell carcinoma.

**Table 4.** Correlation between HMGA2 expression and the clinical pathological features of 60 LSCC patients

Characteristic	All cases	HMGA2 expression		P-value
		High (n = 30)	Low (n = 30)	
Gender				0.284
male	38	17	21	
female	22	13	9	
Age (years)				0.118
< 60	26	10	16	
≥60	34	20	14	
Smoking history				0.390
Nonsmokers	17	7	10	
Current smokers	43	23	20	
Lymph nodes metastasis				0.002*
Negative	32	10	22	
Positive	28	20	8	
TNM Stages				0.002*
I/II	28	8	20	
III/IV	32	22	10	

*P <0.05; LSCC, laryngeal squamous cell carcinoma.

### Silencing of circSHKBP1 restrained the tumorigenesis of LSCC via modulating miR-766-5p/HMGA2 axis

To validate whether circSHKBP1 modulated the tumorigenesis of LSCC via miR-766-5p/HMGA2 axis, cells were transfected with HMGA2 overexpressing vector. The results demonstrated that HMGA2 level in the HMGA2 group was prominently increased in comparison with the control vector group (*P* <0.05), which indicated that HMGA2 was transfected successfully (Figure 5a). The viability of TU686 and AMC-HN-8 cells in the si-circSHKBP1 group was lower than that in the si-NC group, however, compared with the si-circSHKBP1 group, cell viability was obviously facilitated both in the si-circSHKBP1+ miR-766-5p inhibitor group and in the si-circSHKBP1+ HMGA2 group, suggesting that miR-766-5p inhibitor or HMGA2 could effectively eliminate the effect of si-circSHKBP1 on cell viability (Figure 5b). Similarly, miR-766-5p inhibitor or HMGA2 enhanced the abilities of invasion, tube formation and sphere formation that were affected by si-circSHKBP1, which was displayed in Figure 5c-5f. Moreover, si-circSHKBP1 obviously reduced the levels of PCNA, MMP2, VEGFA and OCT4, the effects of which were abrogated by co-transfection with miR-766-5p inhibitor or HMGA2 (Figure 5g). However, the viability and expression levels of PCNA, MMP2, VEGFA and OCT4 were not altered by HMGA2 upregulation in 16-HBE cells (**Supplemental Figure 1D-1 F**). Hence, these results indicated that si-circSHKBP1 restrained the tumorigenesis of LSCC through modulating miR-766-5p/HMGA2 axis.

**Figure 5.** Silencing of circSHKBP1 restrained the tumorigenesis of LSCC by modulating miR-766-5p/HMGA2 axis. (a) Western blotting assay for transfection efficacy of HMGA2 in LSCC cells, *P <0.05, compared with the vector group; (b-f) The influences of si-circSHKBP1/miR-766-5p/HMGA2 on cell viability, invasion, angiogenesis, stem cell-like properties were measured by CCK-8, transwell, angiogenesis, and sphere formation assays, respectively; (g) The protein levels of PCNA, MMP2, VEGFA and OCT4 were determined. *P <0.05, **P <0.01, ***P <0.001. Experiments were conducted in triplicate.

### Silencing of circSHKBP1 suppressed tumorigenesis in vivo

The influences of circSHKBP1 on the tumorigenesis of LSCC were further proved in xenografted mouse models. As presented in Figure 6a-6c, the tumor size and weight of mice were remarkably suppressed in the sh-circSHKBP1 group in contrast to the sh-NC group (*P* <0.01), whereas there was no obvious change about the body weight (*P* >0.05). The levels of circSHKBP1 and HMGA2 in tumor tissues were decreased, while miR-766-5p expression was increased after treatment with sh-circSHKBP1 (*P* <0.05) (Figure 6d). Immunohistochemistry results revealed that the levels of PCNA, MMP2, VEGFA and OCT4 in the sh-circSHKBP1 group were conspicuously decreased in contrast to the sh-NC group (*P* <0.05) (Figure 6e). All the data manifested that downregulation of circSHKBP1 suppressed the tumorigenesis of LSCC *in vivo*.

**Figure 6.** Silencing of circSHKBP1 suppressed the tumorigenesis of LSCC *in vivo*. (a-c) The tumor size, body weight and tumor weight were shown in mice after injection of AMC-HN-8 cells transfected with sh-circSHKBP1 or sh-NC; (d) qRT-PCR assay for levels of circSHKBP1, miR-766-5p and HMGA2 in tumor tissues; (e) Immunohistochemistry method was used to examine levels of HMGA2, PCNA, MMP2, VEGFA and OCT4 in mouse tumor tissues. *P <0.05, **P <0.01, compared with the sh-NC group. Experiments were conducted in triplicate.

## Discussion

To our knowledge, dysregulation of circRNAs is often occurred in various cancers, in which they are deemed as master regulators in disease progression [23]. Noteworthy, previous study has disclosed that circRNA-miRNA-RNA network was involved in the progression of LSCC [24]. Here, our study displayed that circSHKBP1 was highly expressed in LSCC and high level of circSHKBP1 was relevant to poor prognosis. Moreover, silencing of circSHKBP1 restrained the tumorigenesis of LSCC by targeting miR-766-5p/HMGA2 axis, which was demonstrated by cell viability, invasion, angiogenesis and stem cell-like properties.

Previous study has revealed that angiogenesis can offer oxygen and nutrient, followed by modulating tumor development [25]. circRNA has been demonstrated to regulate the angiogenesis of glioma-exposed endothelial cells [26]. Xie et al. [15] disclosed that circSHKBP1 accelerated VEGF expression and angiogenesis. VEGF, a well-known regulator of angiogenesis [27], is released by regulating proteases including MMP2 [28]. Dysregulated circSHKBP1 was observed in numerous cancers [14,15,29], the abnormal expression of circSHKBP1 was exclusively discovered in squamous tumors [30]. However, whether circSHKBP1 was involved in LSCC development has been poorly defined. The current study displayed that circSHKBP1 was up-regulated in LSCC, and si-circSHKBP1 restrained the viability, invasion, angiogenesis, and stem cell-like properties in LSCC. PCNA, a proliferation indicator, is generally utilized to estimate tumorigenesis [31,32]. MMP2 is involved in tumor invasion and angiogenesis [33]. OCT4, a representative marker of cancer stem cells, was highly expressed in LSCC tissues, which led to the carcinogenesis of LSCC [34,35]. CD133 is also an important marker of stem cell-like properties in LSCC [36]. This study demonstrated that si-circSHKBP1 suppressed the levels of PCNA, MMP2, VEGFA, and OCT4 in LSCC. These findings indicated that circSHKBP1 exerted a crucial function in LSCC development.

Emerging evidence clarifies that circRNA acts as a ceRNA to regulate LSCC tumorigenesis [24]. To date, it remains vague about circSHKBP1-associated-ceRNA network in LSCC progression. Recently, miRNA-targeted therapy attracts more and more attention because it plays a critical role in various cancers. In terms of miR-766-5p, it was down-regulated in the patients with glioma and lymphoma, and the level of miR-766-5p might be deemed as a diagnostic indicator in these diseases [37]. In this study, miR-766-5p was down-regulated in LSCC, and LSCC patients with lower miR-766-5p expression had shower overall survival. Previous studies have demonstrated the connection between miR-766-5p and circRNAs. For instance, miR-766-5p suppressed tumor growth *in vivo*, and miR-766-5p inhibitor attenuated the cancer-promoting effects of si-CASC15 in lung cancer [16]. Another study reported that sh-PRKCZ-AS1 restrained lung adenocarcinoma progression by sponging miR-766-5p [17]. However, about the relationship between miR-766-5p and circSHKBP1, it has not been proved yet. This study firstly disclosed that circSHKBP1 was negatively relevant to miR-766-5p, and miR-766-5p inhibitor attenuated the influences of si-circSHKBP1 on LSCC. Thus, miR-766-5p might be a pivotal gene to link the circSHKBP1-associated network in the progression of LSCC.

HMGA2 is a key member of HMGA family, which contains the binding sites of chromosomal DNA and facilitates neoplastic transformation [38,39]. Recent studies pointed out that HMGA2 not only influenced tumor progression but also acted as an indicator to evaluate the efficacy of chemotherapeutic medications [40–44]. Antonio Palumbo et al. [45] proved that HMGA2 was overexpressed in larynx carcinomas. Consistent with this study, we also demonstrated that HMGA2 expression was promoted in LSCC and it facilitated LSCC tumorigenesis. Moreover, we observed that HMGA2 was the target of miR-766-5p, and it could be positively mediated by circSHKBP1 via miR-766-5p. Importantly, overexpression of HMGA2 reversed the functions of si-circSHKBP1 on LSCC development. These findings indicated that circSHKBP1 promoted the tumorigenesis of LSCC by modulating HMGA2 via targeting miR-766-5p. However, the relations among circSHKBP1, miR-766-5p and HMGA2 were not verified by using rescue experiments in animals, this is one of the limitations of our study. We will investigate their relations in animal experiments in the following study.

## Conclusion

In conclusion, circSHKBP1 was firstly disclosed to modulate LSCC tumorigenesis via regulating miR-766-5p/HMGA2 axis. The circSHKBP1/miR-766-5p/HMGA2 network may be deemed as emerging targets for the therapy of LSCC. To make great progress in clinical translation, the upstream factors and more possible targets of circSHKBP1 are still needed to be further explored.

## Supplementary Material

Supplemental Material

## Data Availability

All data during this study are included in this article.
